# MiR-208a-3p functions as an oncogene in colorectal cancer by targeting PDCD4

This article has been retracted.

**DOI:** 10.1042/BSR20181598

**Published:** 2019-04-16

**Authors:** Henglan Wu, Lele Xu, Yaou Chen, Chunfang Xu

**Affiliations:** 1 Department of Nephrology, First Affiliated Hospital of Jiaxing University, Jiaxing,China; 2 Department of Gastroenterology, The First Affiliated Hospital of Soochow University, Suzhou 215200, Jiangsu, China; 3 Department of Critical Care Medicine, Suzhou Municipal Hospital, Suzhou 215200, Jiangsu, China

**Keywords:** Colorectal cancer, micrRNA-208-3p, PDCD4

## Abstract

Accumulating evidences have shown microRNAs (miRNAs) play important roles in the progression of human cancers including colorectal cancer (CRC). However, the biological function and molecular mechanism of miRNAs in CRC still remains to be further investigated. Using microarray, we found and confirmed that miR-208a-3p was up-regulated in CRC tissues. Its high expression was statistically associated with distant metastasis and TNM stage. Functional assays revealed inhibition of miR-208a-3p suppressed proliferation, invasion and migration, and induced cell apoptosis of CRC cells. Moreover, we identified programmed cell death protein 4 (PDCD4), a well-known tumor suppressor, is a direct target of miR-208a-3p. We also found that overexpression of PDCD4 suppressed cell proliferation, invasion, and migration. Importantly, silencing of PDCD4 efficiently abrogated the promoting effects on CRC cells proliferation, invasion, and migration caused by inhibition of miR-208a-3p. Our findings confirmed the oncogenic role of miR-208a-3p via targeting PDCD4 in CRC, identifying miR-208a-3p as a potential diagnosis and therapeutic biomarker for CRC.

## Introduction

Colorectal cancer (CRC) is one of the most commonly diagnosed cancers and the third leading cause of cancer-related deaths worldwide [1]. According to statistics, in China, there are approximately 376300 new CRC cases and 191000 deaths in 2015 [2]. Although much progress that has been made in diagnosis and treatment of CRC in the last decades, CRC remains a highly fatal tumor due to tumor recurrence and distant metastasis [3]. However, the molecular mechanisms underlying these processes are not well understood.

MicroRNAs (miRNAs) are a class of small non-coding RNAs, which negatively regulate gene expression at post-transcription level by binding to the 3′-untranslated region (3′-UTR) of the mRNA of target genes [4,5]. Recently, aberrant expression of miRNAs has been identified as effective tumor biomarkers for CRC diagnosis, or (and) key oncogenes (or tumor suppressor) modulation [6–9]. For example, Ge et al. [10] showed that miR-196a and miR-196b expressions are frequently up-regulated in CRC tissues and to be associated with clinical stages and survival progression. Xu et al. [11] showed that miR-149 plays an important role in suppressing tumor initiation and progression of CRC by directly targeting forkhead box transcription factor FOXM1. Jiao et al. [12] showed that miR-4261 acted as a tumor suppressor and could cause a significant decrease in tumor cell metastasis *in vitro* and tumor growth in a nude mouse xenograft model. These indicate that miRNAs might play a crucial role in the progression of CRC. However, the understanding of the role and function of miRNAs in the CRC is still in the early stage. Likewise, the roles of many other aberrantly expressed miRNAs in CRC development are still unknown.

In the present study, we first examined the expression profile of miRNAs in CRC tissues and investigated the prognostic value of miR-208a-3p in CRC. Moreover, the roles of miR-208a-3p in CRC progression and the underlying molecular mechanisms for miR-208a-3p to promote CRC progression were explored. Our findings suggest that miR-208a-3p may serve a new diagnosis and therapeutic target for CRC treatment.

## Materials and methods

### Clinical specimens

A total of 40 resected tumor tissues and matched tumor-adjacent tissues were obtained from CRC patients with pathologically diagnostic criteria between January 2015 and July 2016 in the First Affiliated Hospital of Soochow University. The clinicopathological data are shown in Table 1. All human samples were collected in accordance with protocols approved by the Ethics Committee of The First Affiliated Hospital of Soochow University, and all patients gave their informed consent prior to surgery. After surgical removal, the tissues were immediately frozen using liquid nitrogen and stored at −80°C. We confirm that the research has been carried out in accordance with the World Medical Association Declaration of Helsinki, and that all subjects provided written informed consents.

**Table 1:** Associations of miR-208a-3p expression with the clinicopathological characteristics of CRC

Clinical parameters	All cases *n*=40	miR-208a-3p expression		*P*-value
		High (25)	Low (15)	
Gender				0.673
Male	15	10	5	
Female	25	15	10	
Age (years)				0.204
≥60	31	21	10	
<60	9	4	5	
Location				0.571
Proximal colon	26	14	12	
Distal colon and rectum	24	11	13	
Tumor size (cm)				0.087
≥5	28	17	11	
<5	22	8	14	
cTNM stage				0.024*
I + II	26	9	17	
III + IV	24	16	8	
Distant metastasis				0.038*
Absent	30	16	14	
Present	10	9	1	
Histological grade				0.414
Well and moderate	32	19	13	
Poorly	8	6	2	
Lymph node metastasis				0.045*
Present	27	14	13	
Absent	13	11	2	

* *P*<0.05.

### Microarray analysis

Total RNA was extracted from three tumor tissues and paired normal colorectal tissues using miRNeasy Mini kit (Qiagen, Valencia, CA, U.S.A.). Purity and quantity of total RNA were evaluated by NanoDrop ND-1000 Spectrophotometry (Thermo Scientific, U.S.A.) and Agilent’s 2100 Bioanalyzer. miRNA microarray profiling was performed as previously described [13]. Data analysis was performed using GeneSpring GX software (Agilent). Finally, the heat map of the 57 microRNAs most obvious differences was created using a method of hierarchical clustering by GeneSpring GX, version 7.3 (Agilent Technologies, California, United States).

### Quantitative real-time polymerase chain reaction

Total RNA was prepared using TRIzol reagent (Invitrogen) according to the manufacturer’s protocol. Purity of RNA was obtained by checking the optical density (OD) 260/280 ratio using a nanodrop spectrophotometer. For miRNA, cDNA was synthesized using a miScript II RT kit (Qiagen, U.S.A.). The reaction was incubated for 24 h at 37°C, 5 min at 95°C to inactivate miScript Reverse Transcriptase Mix, and placed on ice. For mRNA, 1.0 μg of total RNA was reverse transcribed into cDNA using a PrimeScript RT Reagent Kit (Takara Bio, China) in a 20-μl reaction system according to the manufacturer’s protocol. Real-time PCR for miRNA and mRNA were performed on an ABI PRISM 7300 sequence detection system in an SYBR Green I Real-Time PCR kit (Applied Biosystems; Thermo Fisher Scientific, Inc.). The reaction mixtures were incubated at 94°C for 15 min followed by 40 cycles of 95°C for 10 s, 56°C for 30 s, and 70°C for 30 s. Relative quantitation was determined by normalization to U6 and GAPDH. The primers for quantitative real-time polymerase chain reaction (qRT-PCR) analysis were as follows: miR-208a-3p forward primer: 5′-ATAAGACGAGCAAAAAGCTTGT-3′; miR-208a-3p reverse primer: 5′-GGAACGATACAGAGAAGATTAGC-3′; U6 forward primer: 5′-TGCGGGTGCTCGCTTCGCAGC-3′; U6 reverse primer: 5′-CCAGTGCAGGGTCCGAGGT-3′; programmed cell death protein 4 (PDCD4) forward primer: 5′-AAAGGGAAGGTTGCTGGATA-3′, PDCD4 reverse primer: 5′-CAAAGGAACTGTAGATTGTGTGC-3′; GAPDH forward primer: 5′-CGGAGTCAACGGATTTGGTCGTAT-3′, GAPDH reverse primer: 5′-AGCCTTCTCCAGGTGGTGAAGAC-3′. The qRT-PCR assays were performed in triplicate and the change in expression level was calculated using the 2^−ΔΔ*C*^_t_ method [14].

### Cell lines and cultures

The CRC cell lines including HCT116, SW480, SW620, and HT-29 were obtained from the American Type Culture Collection (ATCC, Manassas, VA). A normal human colon mucosal epithelial cell line NCM460 was purchased from Incell Corporation (San Antonio, TX, U.S.A.) and grown in F-12/Ham medium (Gibco) supplemented with 20% FBS, 0.29 g/l glutamine, and 1% penicillin/streptomycin. All cells were grown in a humidified atmosphere of 95% air and 5% CO_2_ at 37°C.

### Cell transfection

The miR-208a-3p mimics, mimics negative control (mimics NC), miR-208a-3p inhibitor, and inhibitor NC were bought from GenePharm (Shanghai, China). The PDCD4 targeted small interfering RNAs (siRNAs) were synthesized and purified by RiboBio Co. (Guangzhou, China). In addition, the coding domain sequences of PDCD4 mRNA were amplified by PCR, and inserted into pcDNA 3.0 vector to enhance its expression (Invitrogen, Grand Island, NY, U.S.A.), named as pcDNA-PDCD4. HCT116 and SW480 cells (1.0 × 10^6^ per well) were seeded and grown overnight in six-well plates. The next day, transfection was performed using Lipofectamine 2000 (Invitrogen; Thermo Fisher Scientific, Inc.) following manufacturer’s instructions. The final concentration of miRNAs was 50 nM and the PDCD4 expression vector was 0.5 μg/ml. The transfected cells were incubated for 6 h, and normal medium was added, then the cells were harvested for further analysis after 48 h.

### Cell viability

The MTT assay was performed to measure cell viability as described before [15]. After transfection, HCT116 and SW480 cells (3 × 10^3^ per well) were seeded in 96-well plates overnight. At different time points (1, 2, or 3 days), 10 μl MTT solution (5 mg/ml; Sigma, U.S.A.) was added to each well, and the plates were incubated at 37°C for another 4 h. Then the absorbance rates were measured at 450 nm using a microplate reader (Infinite M200; Tecan, Austria). All experiments were performed in triplicate.

### Cell apoptosis assay

Cells were harvested 48 h after transfection. HCT116 and SW480 cells were harvested and washed twice with PBS, then the cells were stained with Annexin V and propidium iodide (PI). After incubation at room temperature in the dark for 15 min, cell apoptosis was analyzed on an FACSCalibur flow cytometer (BD Immunocytometry Systems, U.S.A.).

### Cell invasion assays

Cell transwell assay was performed in a 24-well plate with 8-mm pore size chamber inserts (Corning Incorporated, Corning, NY, U.S.A.). For the invasion assays, after transfection, 1 × 10^5^ cells/well were placed into the upper chamber with or without membrane Matrigel (BD Biosciences, Franklin Lakes, San Jose, CA, U.S.A.), respectively. A 500-μl medium containing 15% FBS was added in the lower chamber. After 36 h of incubation at 37°C in 5% CO_2_, the cells on the upper surface of the membrane were removed, and the cells that had moved to the bottom of the chamber were fixed with 100% methanol for 30 min and stained with 0.1% Crystal Violet for 30 min. The stained cells were imaged and counted using an inverted microscope (Olympus Corporation, Tokyo, Japan).

### Wound healing assay

HCT116 and SW480 cells (1 × 10^6^ per well) were plated on to six-well plates and incubated for 24 h at 37°C. After 24-h transfection, the cells were scrapped with a 10-μl pipette tip and replaced with fresh serum-free medium. Initial images were acquired as a reference and, after 24 h, secondary images were taken corresponding to the formerly photographed region. Wound healing was evaluated by measuring the distance of the wounded region with an absence of cells.

### Prediction of miR-208a-3p target mRNAs

TargetScan (http://www.targetscan.org/) and miRanda (http://www.microrna.org) were used to predict the target mRNAs of miR-208a-3p. Those consistently identified by the two databases were regarded as potential target mRNAs.

### Dual-luciferase reporter assay

For dual-luciferase reporter assays, the 3′-UTR of PDCD4 containing miR-208a-3p binding sites were cloned into a pmirGLO dual-luciferase vector (Promega Corporation, Madison, WI, U.S.A.) to generate wild-type (WT) pmirGLO-PDCD4 3′-UTR. The mutant (MUT) 3′-UTR of *PDCD4* gene with miR-208a-3p target sites were generated using a Site-Directed Mutagenesis kit (Agilent Technologies, Inc., Santa Clara, CA, U.S.A.), and cloned into a pmirGLO dual-luciferase vector (Promega Corporation) to generate MUT pmirGLO-PDCD4 3′-UTR. The WT pmirGLO-PDCD4 3′-UTR and MUT pmirGLO-PDCD4 3′-UTR were co-transfected with miR-208a-3p mimics, inhibitor or negative control (NC) by using Lipofectamine 2000 (Invitrogen; Thermo Fisher Scientific, Inc.). Cells were collected 48 h after the transfection, and the luciferase activities were analyzed with the Dual-Luiferase Reporter Assay System (Promega, U.S.A.) according to the manufacturer’s instructions.

### Indirect immunofluorescent assay

After 48 h transfection, miR-208a-3p-transfected or NC cells were fixed for 20 min with 4% paraformaldehyde, and then washed three times with PBS. The cells were subsequently incubated with primary antibody against cleaved caspase 3 (1:1000, cat no. #9664, Cell Signaling Technology Inc.) in PBS at 4°C overnight. After washing three times with PBS, the cells were incubated with FITC–conjugated goat anti-mouse IgG (Sigma, U.S.A.) for 1 h at RT. Finally, the cells were imaged using a Leica AF6000 fluorescent microscope (Leica AF6000, Wetzlar, Germany).

### Western blot analysis

Cells were lysed in the radio immunoprecipitation assay (RIPA) lysis buffer (Beyotime Biotechnology, Shanghai, China), and the protein concentration was measured by using a BCA Protein Assay kit (Pierce, U.S.A.). Total protein samples (30 μg) were analyzed by 8% SDS/PAGE gel and transferred to polyvinylidene difluoride (PVDF) membranes (GE Healthcare, Freiburg, DE) by electroblotting, which were blocked with 5% non-fat dried milk in TBS-T and then probed with rabbit anti-PDCD4 antibody (1:1000, Abcam, U.K.) and mouse anti-β-actin (1:1000, Sigma, U.S.A.). Then the membranes were incubated with horseradish peroxidase (HRP)–conjugated goat anti-rabbit IgG or goat anti-mouse IgG (Boster BioTec, China). Membranes were then detected by using the enhanced chemoluminescence (ECL) system (Clinx Science Instruments, China).

### Statistical analysis

Statistical analysis was performed using the SPSS program (version 18.0; SPSS, Chicago, IL, U.S.A.). Data were presented as mean ± S.D. Student’s *t* test or one-way ANOVA were used to analyze the difference among/between sample groups. Pearson’s correlation analysis was used to evaluate the correlations between the expression of miR-208a-3p and PDCD4. *P*<0.05 was considered as statistically significant.

## Results

### Identification of miRNAs aberrantly expressed in CRC

In order to better understand the role of miRNAs in CRC progression, we performed miRNAs array on CRC tissues and corresponding normal tissues. The miRNA microarray identified 32 miRNAs that were up-regulated in CRC tissues and 25 miRNAs that were down-regulated compared with their matched tumor-adjacent tissues (Figure 1A). Among them, miR-208a-3p is one of the most significantly up-regulated miRNAs and many studies revealed that miR-208a-3p promotes tumorigenicity of various human cancers cells [16–19], but in CRC, the expression and precise function of this miRNA has not been systematically investigated. To confirm the results of the miRNA microarray analysis, qRT-PCR analysis was used to detect the expression of miR-208a-3p in 40 pairs of fresh CRC tissues and its adjacent non-tumor tissues. As shown in Figure 1B, miR-208a-3p expression in CRC tissues was clearly was noteworthy higher than that of the adjacent non-tumor tissues. In addition, miR-208a-3p was also significantly increased in the four CRC cell lines (HCT116, SW480, SW620, and HT-29) compared with that of normal human colon mucosal epithelial cell line NCM460 (Figure 1C). All data suggest that the alteration in miR-208a-3p expressions may be involved in the carcinogenesis of CRC.

**Figure 1:** miR-208a-3p was up-regulated in CRC tissues and cell lines (**A**) Heat map of miRNA profiles represented the significantly regulated miRNAs. The color code in the heat maps is linear, with green as the lowest and red as the highest. The miRNAs that were up-regulated were shown in green to red, whereas the miRNAs that were down-regulated were shown from red to green. (**B**) miR-208a-3p expression was validated by qRT-PCR in CRC tissues and matched tumor-adjacent tissues (*n*=40). *P*< 0.01 vs. adjacent tissue. (**C**) miR-208a-3p expression was measured in four CRC cell lines HCT116, SW480, SW620, and HT-29, and a normal human colon mucosal epithelial cell line NCM460 used as a control by qRT-PCR. Data represent the mean ± S.D. of three independent experiments. **P < 0.01 vs. NCM460 cells.

To determine the clinical values of miR-208a-3p, we used the mean expression level of miR-208a-3p as a cut-off value to divide 40 CRC patients into two groups: miR-208a-3p high expression group and miR-208a-3p low expression group. The relationship between miR-208a-3p expression and clinicpathological features was summarized in Table 1. We found that the high miR-208a-3p expression was associated with distant metastasis, lymph node metastasis, and TNM stage. However, there was no significant association between patients’ gender, age, location, tumor size, and histological grade, and the expression patterns of miR-208a-3p. These results highlighted the potential role of miR-208-3p as a novel diagnosis biomarker.

### Inhibition of miR-208a-3p suppressed cell proliferation and promoted cell apoptosis

To explore the biological functions of miR-208a-3p in CRC cell lines, HCT116 and SW480 cells which have the highest miR-208a-3p level among the four CRC cell lines, were transfected with the miR-208a-3p inhibitor or inhibitor-NC to induce down-regulation of miR-208a-3p expression. As shown in Figure 2A, the expression level of miR-208a-3p in both HCT116 and SW480 cells was significantly decreased after transfection. The effect of miR-208-3p inhibition on cell proliferation was detected by MTT assay. The results showed that cell proliferation was significantly reduced in miR-208a-3p inhibitor group compared with that in control group (Figure 2B,C). Next, we studied the potential mechanism underlying the effect of miR-208a-3p on the CRC cell growth; we used flow cytometry to analyze cell apoptosis in HCT116 and SW480 cells. It was found that miR-208a-3p inhibition markedly promoted the apoptosis portion compared with that in control group (Figure 2D). Finally, the expression of apoptosis related protein, cleaved-caspase 3 was measured by indirect immunofluorescent assay (IFA). The results of IFA showed that miR-208a-3p inhibitor obviously promoted the expression of cleaved caspase 3 compared with control group (Figure 2E). These results suggest that miR-208a-3p inhibitor diminished proliferation partially through inducing cell apoptosis.

**Figure 2:** Inhibition of miR-208a-3p suppressed cell proliferation and promoted cell apoptosis HCT116 and SW480 cells were transfected with the miR-208a-3p inhibitor or inhibitor-NC for 48 h, and then cells were used for analysis. (**A**) Transfection efficiency was assessed by qRT-PCR. (**B,C**) Cell proliferation was measured by MTT assay at indicated times in HCT116 and SW480 cells. (**D**) The apoptosis was detected by flow cytometry. (**E**) The expression of cleaved caspase 3 was measured by IFA. Data represent the mean ± S.D. of three independent experiments. *P < 0.05, **P< 0.01 vs. inhibitor NC.

### Inhibition of miR-208a-3p suppressed cell invasion and migration

Next, we investigated the effects of miR-208a-3p inhibition on CRC cells invasion and migration ability using transwell assays and wound healing assays. The transwell assay revealed that the invaded cell number was significantly reduced in miR-208a-3p inhibitor-transfected cells compared with cells transfected with the NCs (Figure 3A,B). The wound healing assay showed that miR-208a-3p inhibition clearly decreased the cell migration distance compared with cells transfected with the NCs (Figure 3C,D). These data suggest that miR-208a-3p down-regulation acted as a repressor in colorectal cell migration and invasion.

**Figure 3:** Inhibition of miR-208a-3p suppressed cell invasion and migration HCT116 and SW480 cells were transfected with the miR-208a-3p inhibitor or inhibitor-NC for 48 h, and then cells were used for analysis. (**A,B**) Transwell assay was used to evaluate the effect of miR-208a-3p expression on the invasion ability of CRC cells. (**C,D**) Wound healing assay was used to evaluate the effect of miR-208a-3p expression on cell migration capacity. Data represent the mean ± S.D. of three independent experiments. **P< 0.01 vs. inhibitor NC.

### miR-208a-3p directly targets PDCD4 and inhibits its expression

To illustrate the molecular mechanism by which miR-208a-3p functions in CRC, we searched for candidate genes of miR-208a-3p using TargetScan and miRanda databases. Bioinformatics analyses predicted that PDCD4 was a potential target of miR-208a-3p (Figure 4A). Furthermore, qRT-PCR assay was performed to measure the expression levels of PDCD4 in CRC tissues. As shown in Figure 4B, PDCD4 expression level was markedly down-regulated in CRC tissues compared with the matched tumor-adjacent tissues. The correlation between the expression levels of miR-208a-3p and PDCD4 was examined in CRC tissues. Pearson’s correlation analysis suggested that the expression of PDCD4 was significantly inversely correlated with miR-208a-3p expression in CRC tissues (r  = −0.7021, *P*< 0.01, Figure 4C). To further verify this direct targeting, we overexpressed/knocked down miR-208a-3p in HCT116 and SW480 cells and examined the protein levels of PDCD4 using Western blot analysis. We found that up-regulation of miR-208a-3p expression led to a significant decrease in PDCD4 protein level, whereas inhibition of miR-208a-3p resulted in an obvious elevation (Figure 4D).

**Figure 4:** PDCD4 was a direct target of miR-208a-3p (**A**) Schematic of the PDCD4 3′-UTR containing the miR-208a-3p binding sites. (**B**) The relative expression level of PDCD4 was detected by qRT-PCR in CRC tissues and matched tumor-adjacent tissues (*n*=40). *P* < 0.01 vs. Normal group. (**C**) The negative correlation between PDCD4 and miR-208a-3p levels in CRC tissues (r  = −0.7021, *P*< 0.01). Then, HCT116 and SW480 cells were transfected with the miR-208a-3p mimics, mimics-NC, miR-208a-3p inhibitor, or inhibitor-NC for 48 h, and then cells were used for analysis. (**D**) The expression levels of PDCD4 protein was determined by Western blot. (**E**) Relative luciferase activity in HCT116 cells co-transfection with WT or MUT 3′-UTR PDCD4 reporter plasmids and miR-208a-3p or miR-NC. All data are expressed as the mean ± S.D. **P<0.01 vs. mimics NC, ^##^*P*<0.01 vs. inhibitor NC.

To further evaluate whether the PDCD4 is the direct target of miR-208a-3p, we conducted a luciferase reporter assay. The reporter assay showed that miR-208a-3p mimics significantly decreased the luciferase activity of PDCD4 3′-UTR (WT), whereas miR-208a-3p inhibitor increased the luciferase activity (Figure 4E). However, the luciferase activity of the reporter containing the mutant binding site has no obvious change (Figure 4E). These data demonstrated that PDCD4 was a functional target of miR-208a-3p in CRC.

### Overexpression of PDCD4 suppressed CRC cell proliferation and metastasis

Previous study showed that PDCD4 acted as a potent tumor suppressor in various tumors. For example, PDCD4 was found to suppress cancer cell migration through degrading the collagenous substrates in pancreatic tumor [20]. A previous research also showed that overexpression of PDCD4 has been shown to inhibit cell growth and invasion in breast cancer cells [21]. Therefore, we investigated whether the up-regulation of PDCD4 expression has a similar function in CRC. Then pcDNA-PDCD4 or NC plasmids were transfected into HCT116 and SW480 cells. As shown in Figure 5A,B, PDCD4 protein levels were markedly increased in pcDNA-PDCD4-transfected cells than that in cells transfected with the NC or the vector only. Using the transfected cells, MTT, transwell, and wound healing assays were performed to examine the effects of PDCD4 on cell proliferation and invasion. The MTT assay revealed that cell proliferation was significantly inhibited in pcDNA-PDCD4-transfected cells compared with cells transfected with pcDNA-vector (Figure 5C,D). The transwell assay showed that the invaded cell number was significantly reduced in pcDNA-PDCD4-transfected cells compared with cells transfected with pcDNA-vector (Figure 5E,F). The wound healing assay revealed that PDCD4 overexpression clearly decreased the cell migration distance compared with cells transfected with pcDNA-vector (Figure 5G,H). These data suggest that PDCD4 acted as a tumor suppressor in CRC cells.

**Figure 5:** Overexpression of PDCD4 suppressed cell proliferation, invasion, and migration HCT116 and SW480 cells were transfected with the pcDNA-PDCD4 vector or pcDNA3.1 vector for 48 h, and then cells were used for analysis. (**A,B**) Transfection efficiency was assessed by Western blot. Data represent the mean ± S.D. of three independent experiments. **P< 0.01 vs. Blank group (non-treated cells) and pcDNA-vector. (**C,D**) Cell proliferation was measured by MTT assay at indicated times in HCT116 and SW480 cells. (**E,F**) Transwell assay was used to evaluate the effect of PDCD4 expression on the invasive ability of CRC cells. (**G,H**) Wound healing assay was used to evaluate the effect of miR-208a-3p expression on cell migration capacity. Data represent the mean ± S.D. of three independent experiments. *P<0.05, **P< 0.01 vs. pcDNA-vector.

### Down-regulation of miR-208a-3p inhibited CRC cell proliferation, invasion and induced cell apoptosis by targeting PDCD4

Then the question was raised: could miR-208a-3p affect the cellular functions of CRC cells by regulating the expression of PDCD4? To answer it, we knocked down PDCD4 by siRNA (si-PDCD4) in HCT116 and SW480 cells. Compared with control siRNA transfection, si-PDCD4 transfection significantly decreased the expression of PDCD4 protein in both HCT116 and SW480 cells (Figure 6A). Meanwhile, the miR-208a-3p inhibitor-induced increase in PDCD4 protein expression levels was significantly inhibited by transfection with si-PDCD4 (Figure 6B). Moreover, the results showed that the regulation of cell proliferation, apoptosis, migration, and invasion by miR-208a-3p inhibitor transfection were reversed by co-transfection of si-PDCD4 (Figure 6C–F). These data suggest that miR-208a-3p exerts its oncogenic role in CRC at least partially through targeting PDCD4.

**Figure 6:** Down-regulation of miR-208a-3p inhibited CRC cell proliferation, invasion and induced cell apoptosis by targeting PDCD4 HCT116 and SW480 cells were co-transfected with the si-PDCD4 and/or miR-208a-3p inhibitor for 48 h, and then cells were used for analysis. (**A,B**) The protein expression of PDCD4 was measured by Western blot. (**C**) Cell proliferation was measured by MTT assay at indicated times in HCT116 and SW480 cells. (**D**) The apoptosis was detected by flow cytometry. (**E**) Transwell assay was used to evaluate the invasive ability of CRC cells. (**F**) Wound healing assay was used to evaluate the cell migration capacity. Data represent the mean ± S.D. of three independent experiments. *P<0.05, **P<0.01 vs. inhibitor NC; ^##^*P*<0.01 vs. miR-208a-3p inhibitor.

### Overexpression of miR-208a-3p promoted CRC cell proliferation and invasion by down-regulating PDCD4

Next, we investigated whether overexpression of miR-208a-3p promoted CRC cell proliferation and invasion by down-regulating PDCD4. To verify our hypothesis, SW620 and HT29 cells which have the lowest miR-208a-3p level among the four CRC cell lines, were co-transfected with the miR-208a-3p mimics and pcDNA-PDCD4. As shown in Figure 7A, the expression level of PDCD4 was significantly decreased in miR-208a-3p mimics transfected SW620 and HT29 cells, however, after co-transfecting with pcDNA-PDCD4 plasmid the level of PDCD4 significantly increased. Moreover, we found that miR-208a-3p overexpression significantly promoted the cell proliferation, invasion, and migration in both SW620 and HT29 cells, compared with mimics NC group. However, these promoting effects of miR-208a-3p were obviously reversed by PDCD4 overexpression (Figure 7B–D). Collectively, these results suggest that miR-208a-3p regulated CRC cells proliferation, invasion, and migration at least partially through targeting PDCD4.

**Figure 7:** Overexpression of miR-208a-3p promoted CRC cell proliferation and invasion by down-regulating PDCD4 SW620 and HT29 cells were co-transfected with the miR-208a-3p mimics and pcDNA-PDCD4 for 48 h, and then cells were used for analysis. (**A**) The protein expression of PDCD4 was measured by Western blot. (**B**) Cell viability was measured by MTT assay in SW620 and HT29 cells. (**C**) Transwell assay was used to evaluate the invasive ability of CRC cells. (**D**) Wound healing assay was used to evaluate the cell migration capacity. Data represent the mean ± S.D. of three independent experiments. *P<0.05, **P<0.01 vs. mimics NC; ^##^*P*<0.01 vs. miR-208a-3p mimics.

## Discussion

In the present study, miR-208a-3p was up-regulated in human CRC tissues and cell lines, and associated with distant lymph node metastasis and TNM stage of CRC. Further experiments indicated that the effect of miR-208a-3p on CRC cell proliferation, invasion, and migration was mediated by targeting PDCD4. Our results provided new potential biomarkers and targets for CRC diagnosis and treatment.

Accumulating evidence has suggested that miRNAs play a crucial role in the development and progression of CRC with potential diagnostic, prognostic, and therapeutic values in clinical [22,23]. For example, Wang et al. [24] showed that miR-375 was frequently down-regulated in human CRC cell lines and tissues, and overexpression of miR-375 suppressed CRC cell proliferation and colony formation and led to cell cycle arrest. Li et al. [25] demonstrated that miR-139-5p inhibited epithelial–mesenchymal transition (EMT) and enhanced the chemotherapeutic sensitivity of CRC cells by regulating BCL2 expression. In this study, we screened the miRNA expression pattern in CRC tissues and found miR-208a-3p was a CRC-associated miRNA. Further studies demonstrated that miR-208a-3p was commonly up-regulated in CRC tumor tissues and cell lines. Importantly, miR-208a-3p expression was significantly correlated with distant metastasis, lymph node metastasis, and TNM stage. These results indicated that aberrant expression of miR-208a-3p may be crucial for CRC progression. It has been reported that miR-208-3p could participate in the tumorigenesis of pancreatic cancer (PC), human esophageal squamous cell carcinoma (ESCC), and hepatocellular carcinoma (HCC) [16–18]. However, its biological role and molecular mechanism in CRC remains poorly understood. We next investigated the function and potential mechanisms underlying the effect of miR-208a-3p on regulating the biological behavior of CRC cells. Inhibition of miR-208a-3p can suppress CRC cell proliferation, migration and invasion, and induced cell apoptosis, which revealed the crucial role of miR-208-3p in CRC.

PDCD4 is a key protein involved in programmed cell death and has been known as a novel tumor suppressor in several human cancers [20,26,27]. For example, Lankat-Buttgereit et al. [28] showed that PDCD4 basically exerts its function through repressing cell cycle progression at G_1_ stage and PDCD4 loss results in cell cycle acceleration in ovarian cancer. It also has been demonstrated that PDCD4 can induce the expression of cyclin-dependent kinase inhibitors, p21 and p27, resulting in the inhibition of cell cycle progression [29,30]. To date, a set of miRNAs have been confirmed to target PDCD4, such as miR-21 in cervical cancer [31], miR-183-5p in breast cancer [32], and miR-96 in glioma cancer [33]. Although the correlation of miR-208a-3p and PDCD4 has been demonstrated [34], the exact mechanisms of miR-208a-3p/PDCD4 in CRC remain unknown yet. In our study, we demonstrated that PDCD4 was down-regulated in CRC tissues and directly regulated by miR-208a-3p in CRC tissues and cells. Moreover, PDCD4 overexpression significantly inhibited proliferation, invasion, and migration in CRC cells. More importantly, PDCD4 overexpression (inhibition) abrogated the effects of miR-208a-3p mimics (inhibitor), suggesting that PDCD4 mediated, at least in part, the oncogenic effect of miR-208a-3p in CRC cells.

In conclusion, we have provided new evidence suggesting that miR-208a-3p functions as an oncogene by targeting PDCD4 in CRC. Our findings suggest that miR-208a-3p/PDCD4 could be an effective target for the development of effective CRC therapies.

## Abbreviations

Bcl-2: B-cell lymphoma 2
CRC: colorectal cancer
GAPDH: glyceraldehyde 3-phosphate dehydrogenase
IFA: indirect immunofluorescent assay
MUT: mutant-type
NC: negative control
PDCD4: programmed cell death protein 4
qRT-PCR: quantitative real-time polymerase chain reaction
RT: reverse transcription
TBST: Tris-buffered saline with 0.1% Tween 20
TNM: tumor node metastasis
U6: small nuclear RNA U6
WT: wild-type
3′-UTR: 3′-untranslated region
